The article "Research on the Undulatory Motion Mechanism of Seahorse Based on Dynamic Mesh" was published in 2021. Journal: Appl Bionics Biomech.

# Research on the Undulatory Motion Mechanism of Seahorse Based on Dynamic Mesh

**DOI:** 10.1155/2021/2807236

**Published:** 2021-09-20

**Authors:** Xinyu Quan, Ximing Zhao, Shijie Zhang, Jie Zhou, Nan Yu, Xuyan Hou

**Affiliations:** State Key Laboratory of Robotics and System, Harbin Institute of Technology, No. 2 Yikuang Street, Nangang, Harbin City, Heilongjiang Province, China 150080

## Abstract

The seahorse relies on the undulatory motion of the dorsal fin to generate thrust, which makes it possess quite high maneuverability and efficiency, and due to its low volume of the dorsal fin, it is conducive to the study of miniaturization of the driving mechanism. This paper carried out a study on the undulatory motion mechanism of the seahorse's dorsal fin and proposed a dynamic model of the interaction between the seahorse's dorsal fin and seawater based on the hydrodynamic properties of seawater and the theory of fluid-structure coupling. A simulation model was established using the Fluent software, and the 3D fluid dynamic mesh was used to study the undulatory motion mechanism of the seahorse's dorsal fin. The effect of the swing frequency, amplitude, and wavelength of the seahorse's dorsal fin on its propulsion performance was studied. On this basis, an optimized design method was used to design a bionic seahorse's dorsal fin undulatory motion mechanism. The paper has important guiding significance for the research and miniaturization of new underwater vehicles.

## 1. Introduction

With the increasing demand for natural resources in modern society, the speed of exploitation of terrestrial resources is difficult to meet people's needs for material life. The ocean, which accounts for 71% of the entire surface of the earth, has become a treasure trove of resources for all countries. There are not only abundant fishery resources and mineral resources but also sufficient energy resources, such as large oil fields and combustible ice. Whether it is economic or military, the treasure of the ocean is attractive enough, and the rapid development of underwater vehicles will become inevitable. The seahorse relies on the undulatory motion of the dorsal fin to generate thrust, which makes it possess quite high maneuverability and efficiency, and due to its low volume of the dorsal fin, it is conducive to the study of miniaturization of the driving mechanism. This article has carried out research on the undulatory motion mechanism of the seahorse's dorsal fin.

The current research on the seahorse mainly focuses on the following aspects: some focus on the distribution and breeding of seahorse populations in global seas [1–3]; some focus on the evolution of the seahorse, as well as basic biological characteristics and living habits [4, 5]; others focus on the kinematics and dynamics of the seahorse's dorsal and caudal fins [6–10]. In addition, a high-speed camera system is used to study the undulatory motion of the seahorse's dorsal fin [11]; and also, some focus on the study of the physiological structure and the mechanical properties of the muscle of the seahorse's dorsal fin [12].

So far, few studies have been conducted on the undulatory motion mechanism of the seahorse's dorsal fin. The reason is mainly due to the uncertainty of living seahorse's movement, which leads to considerable difficulties in the setup of the experimental device, and this uncontrollable movement will also make it difficult for high-speed cameras to obtain sufficient illumination and focus. In addition, differences between seahorse's species, between different genders, and between different individuals will hinder systematic and reproducible research. There are so many difficulties in living animal experiments, so many scholars usually manufacture bionic prototypes for mechanism research. This method can solve the above-mentioned problems, but the prototype dorsal fin is difficult to achieve the swing amplitude and frequency like a living seahorse, and the difficulty in manufacturing and control causes the experimental results to be inaccurate. In addition to physical experiments, simulation can also be used to study the mechanism of seahorse's movement. However, due to insufficient computer computing power and other reasons, early simulations were mainly two-dimensional plane simulations, which were difficult to directly explore the movement mechanism. Nowadays, the computing power is greatly improved. Compared with physical experiments, fluid-structure coupling simulation can improve the efficiency of experiments and reduce the cost of making prototypes. At the same time, it can reduce the impact of the uncontrollable motion of the living seahorse on the experiment, and it is beneficial to the systematic and repeatable research [13].

Based on the theory of fluid-structure interaction, this paper uses Fluent software to construct a dynamic model of the interaction between the seahorse dorsal fin and seawater. The influence of the different swing frequency, wavelength, and amplitude of the dorsal fin on the undulatory motion of the seahorse's dorsal fin was analyzed, which provide important support for the research on the undulatory motion mechanism of the seahorse's dorsal fin. On this basis, an optimal design method was used to design a seahorse-like dorsal fin wave motion mechanism, which has important guiding significance for the development of new underwater vehicle research and the miniaturization of the vehicle.

## 2. Materials and Methods

### 2.1. Physical Model

The seahorse's dorsal fin is composed of fin rays and fin membrane. The length of adult seahorse's dorsal fin is generally between 3 and 25 mm, and the number of fin rays is between 10 and 30. Some types of seahorse are shown in Figure 1 [14], and the number of fins and dorsal fin length of some types of seahorse are shown in Table 1.

The common perpendicular of the fins is defined as the *z*-axis, and this direction is called the chord direction. The *y*-axis is perpendicular to the *z*-axis and straight down, and this direction is called the span direction. Finally, according to the right-hand spiral, determine the *x*-axis direction. The coordinate system is shown in Figure 2. Points on the dorsal fin of the seahorse approximately rotate around the *z*-axis. For the real seahorse's dorsal fin swinging, its swing amplitude should change with the *z*-axis position. In order to simplify the model, it is considered that the swing amplitude does not change with the *z*-axis position.

The kinematics equation of the dorsal fin is

(1) $$\begin{array}{c} \begin{array}{c} r\in \left[0,l\right],\\ z\in \left[0,L\right],\\ \theta =\frac{\pi }{2}+A\sin\left(2\pi ft+\frac{2\pi z}{\lambda }\right),\\ x=r\cos\left(\theta \right),\\ y=r\sin\left(\theta \right), \end{array} \end{array}$$

where *l* is the fin length, *L* is the total length of the dorsal fin, *A* is the swing amplitude, *f* is the swing frequency, *λ* is the swing wavelength, and *t* is time.

First, calculate the coordinates of a large number of points on the dorsal fin in excel. Then, import them to Solidworks to generate a point cloud, as shown in Figure 3(a). Through surface treatment, the physical model of the dorsal fin is obtained as shown in Figure 3(b).

### 2.2. Fluid-Structure Coupling Dynamics Modelling

In order to obtain the dynamic model of the seahorse's dorsal fin, the dynamic equation of the seahorse's dorsal fin needs to be established first. First, establish two coordinate systems, one of which is fixedly connected to the seahorse's dorsal fin and is called the coordinate system O′. And the other is an inertial coordinate system which is called the coordinate system O. The two coordinate systems coincide at the initial moment.

The position of the origin of the coordinate system O′ is given by:

(2) $$\begin{array}{c} \begin{array}{c} a=a_{0}+\int v_{x}dt,\\ b=b_{0}+\int v_{y}dt,\\ c=c_{0}+\int v_{z}dt, \end{array} \end{array}$$

where *a*, *b*, *c* is the position of the origin of the coordinate system O′ in the coordinate system O. *a*_0_, *b*_0_, *c*_0_ is the initial position of the origin of the coordinate system O′ in the coordinate system O. *v*_*x*_, *v*_*y*_, *v*_*z*_ is the speed of origin of the coordinate system O′ along the *x*-, *y*-, and *z*-axes in the coordinate system O.

The relationship between Euler angle change rate and angular velocity is given by:

(3) $$\begin{array}{c} \left[\begin{array}{c} \alpha^{\prime }\\ \phi^{\prime }\\ \theta^{\prime } \end{array}\right]=\left[\begin{array}{ccc} 1 & \tan\phi \sin\alpha & \tan\phi \cos\alpha \\ 0 & \cos\alpha & -\sin\alpha \\ 0 & \sin\alpha /\cos\phi & \cos\alpha /\cos\phi \end{array}\right]\cdot \left[\begin{array}{c} \omega_{x}\\ \omega_{y}\\ \omega_{z} \end{array}\right]. \end{array}$$

Then, we can get the Euler angle by:

(4) $$\begin{array}{c} \begin{array}{c} \alpha =\alpha_{0}+\int \omega_{x}dt+\int \tan\phi \sin\alpha \cdot \omega_{y}dt+\int \tan\phi \cos\alpha \cdot \omega_{z}dt,\\ \phi =\phi_{0}+\int \cos\alpha \cdot \omega_{y}dt-\int \sin\alpha \cdot \omega_{z}dt,\\ \theta =\theta_{0}+\int \frac{\sin\alpha \cdot \omega_{y}}{\cos\phi }dt+\int \frac{\cos\alpha \cdot \omega_{z}}{\cos\phi }dt, \end{array} \end{array}$$

where *α*, *ϕ*, *θ* is the Euler angle of the coordinate system O′. *α*_0_, *ϕ*_0_, *θ*_0_ is the initial Euler angle of the coordinate system O′. *ω*_*x*_, *ω*_*y*_, *ω*_*z*_ is the angular velocity of the coordinate system O′.

The speed in formula (2) is obtained by:

(5) $$\begin{array}{c} \overset{⟶}{v}={\overset{⟶}{v}}_{0}+\int \frac{\overset{⟶}{F}}{m}dt+\int \frac{\overset{⟶}{M}}{I_{c}}\times {\overset{⟶}{r}}_{\text{c}}dt \end{array}$$

where ${\overset{⟶}{v}}_{0}$ is the initial velocity of the origin of the coordinate system O′ in the coordinate system O. $\overset{⟶}{F}$ is the resultant external force on the dorsal fin. *m* is the total mass of the dorsal fin. $\overset{⟶}{M}$ is the resultant moment of the dorsal fin. *I*_*c*_ is the moment of inertia with the center of rotation as the axis of rotation. ${\overset{⟶}{r}}_{\text{c}}$ is the distance between the origin of the coordinate system O′ and the center of mass.

The angular velocity in formula (4) is solved by

(6) $$\begin{array}{c} \overset{⟶}{\omega }={\overset{⟶}{\omega }}_{0}+\int \frac{\overset{⟶}{M}}{I_{c}}dt, \end{array}$$

where ${\overset{⟶}{\omega }}_{0}$ is the initial angular velocity of the origin of the coordinate system O′.

The position of any point on the dorsal fin in the coordinate system O is given by:

(7) $$\begin{array}{c} \overset{⟶}{r}=H\left(t\right)*{\overset{⟶}{r}}_{0}\left(t\right), \end{array}$$

where *H*(*t*) is the coordinate transformation matrix. ${\overset{⟶}{r}}_{0}\left(t\right)$ is the position of any point on the dorsal fin in the coordinate system O′.

In order to obtain the required force parameter in the dynamic equation, the N-S (Navier-Stokes) equation under turbulent flow is used to solve it. For incompressible fluids, the N-S equation turns to:

(8) $$\begin{array}{c} \begin{array}{c} f_{x}-\frac{1}{\rho }\frac{\partial p}{\partial x}+v\nabla^{2}v_{x}=\frac{dv_{x}}{dt},\\ f_{y}-\frac{1}{\rho }\frac{\partial p}{\partial y}+v\nabla^{2}v_{y}=\frac{dv_{y}}{dt},\\ f_{z}-\frac{1}{\rho }\frac{\partial p}{\partial_{z}}+v\nabla^{2}v_{z}=\frac{dv_{z}}{dt}, \end{array} \end{array}$$

where *f*_*x*_, *f*_*y*_, and *f*_*z*_ are the mass force components of unit mass fluid in *x*, *y*, and *z* directions. *v*_*x*_, *v*_*y*_, and *v*_*z*_ are the velocity components of the fluid in the *x*, *y*, and *z* directions. *p* is relative pressure. *v* is the kinematic viscosity of the fluid.

The continuity equation for viscous fluid is given by:

(9) $$\begin{array}{c} \nabla \cdot \nu =0. \end{array}$$

There are three existing turbulence numerical simulation methods: Direct Numerical Simulation (DNS), Reynolds Average Navier-Stokes(RANS), and Large Eddy Simulation (LES). RANS is the application of statistical theory of turbulence, which is the simulation method commonly used in engineering. Usually based on Boussinesq's eddy viscosity hypothesis, the zero equation, one equation, or two equations are introduced to close the equation. The zero-equation model has a common shortcoming, that is, the turbulence viscosity coefficient only depends on the local flow parameters, and has nothing to do with the flow elsewhere, which is inconsistent with experimental observations. On this basis, a one-equation model and two-equation model were developed. Among the two-equation model, the SST model has certain accuracy and consumes limited computing resources and has higher calculation accuracy for near-wall surfaces compared to the other two-equation models. Therefore, the SST model is used in this project.

### 2.3. Simulation Model

Use the grid processing software ICEM to mesh the computing space. The area near the fin surface needs to be focused, so the density of mesh nodes near the fin surface increases. The height of the first cell perpendicular to the body surface is 0.05 mm. This height is chosen to make the *y*+ of most of the cells in contact with the body surface fall within the effective range of the standard wall function. At the same time, considering the calculation speed, take the outer division step of the model as 0.1 mm, and the model is shown in Figure 4.

Import the ICEM file into Fluent, and set the seawater parameters according to the seahorse's living environment, and then, you can simulate the undulatory motion process of the seahorse's dorsal fin under different conditions. Set the model boundary parameters as shown in Table 2, and the Fluent simulation preset parameters as shown in Table 3.

The undulatory motion of the seahorse's dorsal fin is controlled by using Fluent UDF. In the numerical calculation process, the instantaneous force acting on the dorsal fin is obtained by integrating the fin surface pressure and shear stress.

## 3. Results and Discussion

### 3.1. Simulation Process

Import the Fluent calculation results into CFD POST for postprocessing, and then, we can get the flow field distribution at any time. Take 1 Hz frequency, 200 mm wavelength, and *π*/5 swing amplitude for qualitative explanation. The pressure distribution on the surface of the dorsal fin in 0.25 s, 0.5 s, 0.75 s, and 1 s is shown in Figure 5.

It can be clearly seen from Figure 5 that one side of the surface of the dorsal fin that pushes the water flow is a high-pressure area, and the other side is a low-pressure area.

Take a section as shown in Figure 6 to obtain the flow field pressure distribution of the section, as shown in Figure 7.

It can be seen more clearly from Figure 7 that one side of the fin along the wave propagation direction is a high-pressure area, and the other side is a low-pressure area. The pressure difference between the two sides results in the generation of forces in the *x* and *z* directions. Since the dorsal fin of this example is composed of two complete sine waves, the forces generated in the *x* direction cancel each other out. Take another section as shown in Figure 8 to obtain the flow field pressure distribution of the section, as shown in Figure 9.

It can be seen from Figure 9 that when the dorsal fin ray swings, due to the pressure difference between the upper and lower fins, a force in the negative direction of the *y*-axis is generated.

### 3.2. The Effect of Dorsal Fin Swing Frequency on Propulsion

Use Fluent to simulate the five swing frequencies of 1 Hz, 10 Hz, 35 Hz, 50 Hz, and 100 Hz. The wavelengths are all 200 mm, and the swing amplitudes are all *π*/5. Record the force of the dorsal fin in *x*, *y*, and *z* directions, respectively, and perform curve fitting in matlab. Since the force scatter diagram has not stabilized in the first few periods, the third and fourth period scatter diagrams are selected for fitting. Since the minimum frequency of 1 Hz and the maximum frequency of 100 Hz are too far apart, the abscissa is set to time multiplied by the frequency of the corresponding working condition, in order to show the difference of different working conditions more clearly and intuitively.

By using a custom function *f*(*x*) = *a*sin(2*πbx* + *c*) + *d* to curve-fit the force data of the dorsal fin at different swing frequencies in the *x* direction, the following results are obtained.

It can be clearly seen from Figure 10(a) that as the frequency increases, the average force *d* and the fluctuation amplitude *a* in the *x* direction both increase. It can be seen from Table 4 that the approximate sinusoidal frequency of the force in the *x* direction is basically the same as the swing frequency of the dorsal fin, and the phase is also basically the same. From Figure 10(b), the fluctuation amplitude *a* and frequency *f* can be better fitted with a quadratic function, and the relationship between the amplitude and frequency of the force fluctuation in the *x* direction of the dorsal fin can be obtained by:

(10) $$\begin{array}{c} F_{x\_\text{amplitude}}=-0.02467\times {\left(f+8.105\right)}^{2}+3.93. \end{array}$$

However, in Figure 10(c), the average force *d* does not change much after 35 Hz.

By using a custom function *f*(*x*) = *a*sin(2*πbx* + *c*) + *d* to curve-fit the force data of the dorsal fin at different swing frequencies in the *y* direction, the following results are obtained.

It can be clearly seen from Figure 11(a) that as the frequency increases, the average force *d* and the fluctuation amplitude *a* in the *y* direction both increase significantly. It can be seen from Table 5 that the approximate sinusoidal frequency of the force in the *y* direction is twice the swing frequency of the dorsal fin, and the phase difference is approximately *π*/2. From Figure 11(b), the amplitude of fluctuation *a* and frequency *f* can be better fitted with a quadratic function, and the relationship between the amplitude of the force fluctuation in the *y* direction of the dorsal fin and the frequency can be obtained by:

(11) $$\begin{array}{c} F_{y\_\text{amplitude}}=-0.02735\times {\left(f+0.5421\right)}^{2}+0.2775. \end{array}$$

From Figure 11(c), the average force *d* and frequency *f* can also be better fitted with a quadratic function, and the relationship between the average force in the *y* direction of the dorsal fin and the frequency can be obtained by:

(12) $$\begin{array}{c} F_{y\_\text{average}}=-0.2353\times {\left(f-0.1594\right)}^{2}-0.3479 \end{array}$$

(13) $$\begin{array}{c} F_{y\_average}=-0.2353\times {\left(f-0.1594\right)}^{2}-0.3479 \end{array}$$

By using a custom function *f*(*x*) = *a*sin(2*πbx* + *c*) + *d* to curve-fit the force data of the dorsal fin at different swing frequencies in the *z* direction, the following results are obtained.

It can be clearly seen from Figure 12(a) that as the frequency increases, the average force *d* and the fluctuation amplitude *a* in the *z* direction both increase significantly. It can be seen from Table 6 that the approximate sinusoidal frequency of the force in the *z* direction is twice the swing frequency of the dorsal fin, and the phase is basically the same. From Figure 12(b), the fluctuation amplitude *a* and frequency *f* can be better fitted with a quadratic function, and the relationship between the amplitude of the force fluctuation in the *z* direction of the dorsal fin and the frequency can be obtained by

(14) $$\begin{array}{c} F_{z\_\text{amplitude}}=-0.05819\times {\left(f+0.1248\right)}^{2}+0.07337. \end{array}$$

From Figure 12(c), the mean force *d* and frequency *f* can also be better fitted with a quadratic function, and the relationship between the mean force in the *z* direction of the dorsal fin and the frequency can be obtained by:

(15) $$\begin{array}{c} F_{z\_\text{average}}=-0.4687\times {\left(f+0.01611\right)}^{2}+0.386 \end{array}$$

In summary, the average force and fluctuation amplitude in each direction increase with the increase of frequency, and the average force and fluctuation amplitude in the *y* and *z* directions have a quadratic relationship with frequency. The amplitude of the force fluctuation in the *x* direction also has a quadratic relationship with the frequency, but the average value of the force in the *x* direction does not change much after 35 Hz. In reference [15], the authors presented an experimental investigation of flexible panels actuated with heave oscillations at their leading edge. Results were presented from kinematic video analysis, particle image velocimetry, and direct force measurements. They draw the conclusion “The magnitudes of both signals (net thrust and power) increase with heaving frequency, as expected.” And they gave the net thrust and power curves of different frequencies as Figure 13. It can be seen that as the frequency increases, the net thrust gradually increases, and it becomes an approximate sine function in the swing period, which verifies the correctness of the simulation in this study.

### 3.3. The Influence of the Swing Wavelength of the Dorsal Fin on the Propulsion Force

Since the total length of the dorsal fin is 400 mm, in order to minimize the force fluctuations in the *x* direction, an integer number of traveling waves should be selected for the entire dorsal fin. Therefore, Fluent is used to simulate the three swing frequencies of 400 mm, 200 mm, and 133 mm, respectively. The frequencies are all 10 Hz, and the swing amplitudes are all *π*/5. Record the force of the dorsal fin in *x*, *y*, and *z* directions, respectively, and perform curve fitting in matlab. Since the force scatter diagram has not stabilized in the first few periods, the third and fourth period scatter diagrams are selected for fitting.

By using a custom function *f*(*x*) = *a*sin(2*πbx* + *c*) + *d* to curve-fit the force data of the dorsal fin at different swing wavelengths in the *x* direction, the following results are obtained.

It can be clearly seen from Figure 14 and Table 7 that as the wavelength increases, the average force *d* in the *x* direction increases. When the swing wavelength is 400 mm, reducing the wavelength can significantly suppress the fluctuation amplitude *a* of the force in the *x* direction. But after the wavelength of 200 mm, the influence of decreasing the wavelength on the amplitude *a* of the force fluctuation in the *x* direction is greatly reduced. The approximate sinusoidal frequency of the force in the *x* direction is basically the same as the swing frequency of the dorsal fin, and the phase changes with wavelength.

By using a custom function *f*(*x*) = *a*sin(2*πbx* + *c*) + *d* to curve-fit the force data of the dorsal fin at different swing wavelengths in the *y* direction, the following results are obtained.

It can be seen from Figure 15 and Table 8 that the average force *d* in the *y* direction increases significantly with the increase of the swing wavelength, but the fluctuation amplitude *a* hardly changes.

By using a custom function *f*(*x*) = *a*sin(2*πbx* + *c*) + *d* to curve-fit the force data of the dorsal fin at different swing wavelengths in the *z* direction, the following results are obtained.

It can be seen from Figure 16 and Table 9 that the mean value *d* of the force in the *z* direction increases significantly with the increase of the swing wavelength, but the fluctuation amplitude *a* hardly changes.

Based on the analysis of the force in the above three directions, it can be seen that when the wavelength is between 400 mm and 200 mm, as the wavelength decreases, the *x* direction fluctuation of the dorsal fin is significantly suppressed while below 200 mm, the impact is small. At the same time, as the wavelength increases, the mean value of the force in the *y* and *z* directions increases significantly, but the fluctuation range is almost unchanged.

### 3.4. The Influence of the Swing Amplitude of the Dorsal Fin on the Propulsion Force

Use Fluent to simulate the three swing amplitudes, the frequency is 10 Hz, and the wavelength is 200 mm. Record the force of the dorsal fin in *x*, *y*, and *z* directions, respectively, and perform curve fitting in matlab. Since the force scatter diagram has not stabilized in the first few periods, the third and fourth period scatter diagrams are selected for fitting.

By using a custom function *f*(*x*) = *a*sin(2*πbx* + *c*) + *d* to curve-fit the force data of the dorsal fin at different swing amplitudes in the *x* direction, the following results are obtained.

From Figure 17 and Table 10, it can be seen that the swing amplitude has little effect on the force in the *x* direction. No matter how the swing amplitude changes, the average force *d* in the *x* direction fluctuates near the 0 line, and the fluctuation amplitude *a* is relatively small. The approximate sinusoidal frequency of the force in the *x* direction is basically the same as the swing frequency of the dorsal fin, and the phase is also basically the same.

By using a custom function *f*(*x*) = *a*sin(2*πbx* + *c*) + *d* to curve-fit the force data of the dorsal fin at different swing amplitudes in the *y* direction, the following results are obtained.

It can be seen from Figure 18 that as the swing amplitude increases, the average force *d* and the fluctuation amplitude *a* in the *y* direction both increase. It can be seen from Table 11 that the approximate sinusoidal frequency of the force in the *y* direction is twice the swing frequency of the dorsal fin, and the phase difference is *π*/2.

By using a custom function *f*(*x*) = *a*sin(2*πbx* + *c*) + *d* to curve-fit the force data of the dorsal fin at different swing amplitude in the *z* direction, the following results are obtained.

It can be seen from Figure 19 that as the swing amplitude increases, the average force *d* in the *z* direction and the fluctuation amplitude *a* both increase. It can be seen from Table 12 that the approximate sinusoidal frequency of the force in the *z* direction is twice the swing frequency of the dorsal fin, and the phase is the same.

In summary, the average value of the force in each direction increases with the increase of the swing amplitude, but the influence on the force in the *x* direction is negligible. At the same time, the increase of the swing will cause the fluctuation of the force to increase.

### 3.5. Design of Undulatory Motion Mechanism Imitating Seahorse's Dorsal Fin

In order to realize that adjacent fins oscillate with a fixed phase difference, a crank-rocker mechanism driven by a crankshaft is designed, as shown in Figure 20.

A crankshaft is composed of a left part, a right part, and a plurality of middle parts, as shown in Figure 21. The left part has two protruding ends, the left of which is in the center while the right one with eccentricity. There is a shaft flat position on the right-side extension to match the middle part. An eccentric hole on the left side of the middle part is matched with the left part, and an eccentric shaft on the right side is matched with the next middle part. There is also a flat shaft position, and there is a 45° phase difference between the left hole and the right shaft, which makes adjacent fins produce a fixed phase difference. The right part also has an eccentric hole to fit with the middle part, and a concentric shaft on the right is connected to the motor. When making crankshaft parts, consider hollowing out the middle disc to reduce the moment of inertia.

The comprehensive problem of the function mechanism means that the functional relationship between the input and output angles corresponding to the rocker and the crank is required to be as close as possible to the given function *ψ* = *f*(*φ*). The comprehensive theory of the mechanism proves that the kinematics of the crank-rocker mechanism has nothing to do with the actual length of the rod, but only with the shape of the mechanism, that is, the relative length between the rods. Let us set the relative length of the crankshaft as *l*_1_ = 1. The relative length of the connecting rod is *l*_2_. The relative length of the pendulum is *l*_3_. The relative length of the frame is *l*_4_. And the initial angle of the crankshaft and the swing lever is *φ*_0_, *ψ*_0_, so there are 5 variables. Therefore, at most five sets of corresponding angular positions can be accurately met. If the organization is required to best approximate the expected function in more positions, the optimal synthesis method can be used. In the optimization design of the kinematics of the planar four-bar linkage, the objective function is generally established according to the kinematics parameters of the mechanism. For example, the movement realized by a four-bar linkage mechanism is an input-output angular function derived from the geometric relationship of the mechanism's movement, and it is required to have the smallest deviation from a given function within a certain range of motion. In the optimization design of linkage mechanism dynamics, it is relatively simple to use the pressure angle and transmission angle in the mechanism as important indicators for the motion analysis and dynamic analysis of the mechanism. In order to obtain good transmission performance and increase the reliability of the mechanism, it is necessary to select the best mechanism dynamics parameters so that the maximum pressure angle is the smallest or the minimum transmission angle is the largest during the movement of the mechanism. In this project, the crank angle is required to be at any position in a circle, that is, when *φ* = *φ*_0_ ~ (*φ*_0_ + 2*π*), the output angle of the rocker is as close to the function *ψ* = *ψ*_0_ + *π*/5(sin(*φ* − *φ*_0_ − *π*/2) + 1) as possible. Assuming that the initial position angles of the crank and the joystick *φ*_0_, *ψ*_0_ correspond to the input and output angles when the joystick is in the right extreme position. In this way, *φ*_0_,  *ψ*_0_ is no longer an independent variable, so there are three relative lever length variables left. Since the three-dimensional search is more complicated and time-consuming, it is assumed that the relative length of the rack is *l*_4_ = 15. Take the relative length of the connecting rod *l*_2_ and the relative length of the rocker *l*_3_ as design variables.

The crank-rocker mechanism is in accordance with the corresponding relationship between the input and output angles between the driving crank and the driven rocker. The independent parameters include the relative length of the rod *l*_2_/*l*_1_,  *l*_3_/*l*_1_, and *l*_4_/*l*_1_ and the initial angular positions of the crank and the rocker *φ*_0_ and *ψ*_0_. As shown in Figure 22, assume that the acute angle between the crank and the rocker and the frame when the pendulum reaches the right limit position is taken as the initial position angle *φ*_0_ and *ψ*_0_. Due to the geometric relationship of the right limit position, the crank and the connecting rod are collinear, so the two initial angles can be determined according to the geometric relationship of the initial position.

(16) $$\begin{array}{c} \psi_{0}=a\cos\frac{{\left(l_{1}+l_{2}\right)}^{2}-l_{3}^{2}-l_{4}^{2}}{2\left(l_{1}+l_{2}\right)l_{4}} \end{array}$$

(17) $$\begin{array}{c} \psi_{0}=a\cos\frac{{\left(l_{1}+l_{2}\right)}^{2}-l_{3}^{2}-l_{4}^{2}}{2l_{3}l_{4}} \end{array}$$

Therefore, the two initial angles can be expressed by other rod lengths and are no longer independent parameters. According to the above assumption, the crank length is the unit length *l*_1_ = 1. Frame length is *l*_4_ = 15. Therefore, the length of the connecting rod *l*_2_ and the length of the rocker *l*_3_ are selected as design variables $X=\left[\begin{array}{c} l_{2}\\ l_{3} \end{array}\right]=\left[\begin{array}{c} x_{1}\\ x_{2} \end{array}\right]$. This turns into a two-dimensional optimization design problem.

Taking the least square deviation of the output angle of the mechanism as the design goal, the given function and the actual function are discretized, and the discrete deviation function is obtained. The sum of the discrete deviation functions is used as the objective function, as shown in

(18) $$\begin{array}{c} \min f\left(X\right)=\overset{\infty }{\underset{i=0}{\sum }}{\left(\psi_{i}-\psi_{si}\right)}^{2}, \end{array}$$

where *ψ*_*i*_ is the expected output angle and *ψ*_*si*_ is the actual output angle.

According to the given functional relationship and the corresponding relationship between the two initial angles, the output angle expression can be obtained by

(19) $$\begin{array}{c} \psi_{i}=\psi_{0}+\frac{\pi }{5}\left(\sin\left(\varphi -\varphi_{0}-\frac{\pi }{2}\right)+1\right), \end{array}$$

(20) $$\begin{array}{c} \varphi_{i}=\varphi_{0}+\frac{\pi }{2}\times \frac{i}{s}\left(i=0,1,2,\cdots ,s\right) \end{array}$$

where *s* is the uniform number of discrete points of the crank angle *φ* in the interval *φ*_0_ ~ (*φ*_0_ + 2*π*) and *i* is the serial number of each discrete point. The actual output angle expression can be determined according to the geometric relationship of the movement of the mechanism, as shown in Figure 23.

(21) $$\begin{array}{c} \psi_{si}=\left\{\begin{array}{c} \pi -\alpha_{i}-\beta_{i},\\ \pi -\alpha_{i}+\beta_{i}, \end{array}\right.\begin{array}{c} \left(0<\varphi_{i}⩽\pi \right),\\ \left(\pi <\varphi_{i}⩽2\pi \right). \end{array} \end{array}$$

Among them, in Δ*BDC* and Δ*ABD*, applying the law of cosines, we can get

(22) $$\begin{array}{c} \left\{\begin{array}{c} \alpha_{i}=\text{acos}\frac{r_{i}^{2}+x_{2}^{2}-x_{1}^{2}}{2r_{i}x_{2}},\\ \beta_{i}=\text{acos}\frac{r_{i}^{2}+l_{4}^{2}-l_{1}^{2}}{2l_{4}r_{i}},\\ r_{i}=\sqrt{l_{4}^{2}+l_{1}^{2}-2l_{1}l_{4}\cos\varphi_{i}}. \end{array}\right. \end{array}$$

In order to make the transmission performance of the mechanism better, the minimum transmission angle of the mechanism *γ*_min_ ≥ 45° and the maximum transmission angle of the mechanism *γ*_max_ ≤ 135°. When the crank and the frame are collinear, the mechanism has the minimum or maximum transmission angle, as shown in Figure 24. When the mechanism is in these two positions, the law of cosines can be used to obtain by:

(23) $$\begin{array}{c} \left\{\begin{array}{c} \cos\gamma_{\min}=\frac{x_{1}^{2}+x_{2}^{2}-{\left(l_{4}-l_{1}\right)}^{2}}{2x_{1}x_{2}}⩽\cos45^{{}^{\circ}},\\ \cos\gamma_{\max}=\frac{x_{1}^{2}+x_{2}^{2}-{\left(l_{4}+l_{1}\right)}^{2}}{2x_{1}x_{2}}⩾\cos135^{{}^{\circ}}. \end{array}\right. \end{array}$$

After sorting, get the constraint equation:

(24) $$\begin{array}{c} \left\{\begin{array}{c} g_{1}\left(X\right)=x_{1}^{2}+x_{2}^{2}-2\cos45^{{}^{\circ}}x_{1}x_{2}-{\left(15-1\right)}^{2}⩽0,\\ g_{2}\left(X\right)=-x_{1}^{2}-x_{2}^{2}+2\cos135^{{}^{\circ}}x_{1}x_{2}-{\left(15+1\right)}^{2}⩽0. \end{array}\right. \end{array}$$

According to the condition of the sum of the rod lengths of the crank connecting rod (in the crank-rocker mechanism, the crank is the shortest rod, and the sum of the length of the shortest rod and the longest rod is not greater than the sum of the lengths of the other two rods), the constraint conditions are obtained after sorting out:

(25) $$\begin{array}{c} \left\{\begin{array}{c} l_{2}⩾l_{1},\\ l_{3}⩾l_{1},\\ l_{2}+l_{3}⩾l_{1}+l_{4},\\ l_{3}+l_{4}⩾l_{1}+l_{2},\\ l_{2}+l_{4}⩾l_{1}+l_{3}, \end{array}\right.\begin{array}{c} g_{3}\left(X\right)=l_{1}-x_{1}⩽0,\\ g_{4}\left(X\right)=l_{1}-x_{2}⩽0,\\ g_{5}\left(X\right)=\left(l_{4}+l_{1}\right)-x_{1}-x_{2}⩽0,\\ g_{6}\left(X\right)=x_{1}-x_{2}-\left(l_{4}-l_{1}\right)⩽0,\\ g_{7}\left(X\right)=-x_{1}+x_{2}-\left(l_{4}-l_{1}\right)⩽0. \end{array} \end{array}$$

Draw the constrained planning area of the optimal design problem, as shown in Figure 25. It can be seen from the figure that the constraint condition of the sum of the rod length of the crank is a nonfunctional constraint, and the effective constraint is the constraint condition of the mechanism transmission angle *g*_1_(*X*) ⩽ 0 and *g*_2_(*X*) ⩽ 0. The area enclosed by them is the feasible region of the two design parameters.

In summary, the mathematical model of the optimization problem is

(26) $$\begin{array}{c} \left\{\begin{array}{c} \min f\left(X\right)=\min\underset{i=0}{\sum }{\left(\psi_{i}-\psi_{ii}\right)}^{2}\;X\in D,\\ X=\left[\begin{array}{c} l_{2}\\ l_{3} \end{array}\right]=\left[\begin{array}{c} x_{1}\\ x_{2} \end{array}\right],\\ g_{1}\left(X\right)=x_{1}^{2}+x_{2}^{2}-2\cos45^{{}^{\circ}}x_{1}x_{2}-{\left(l_{4}-l_{1}\right)}^{2}⩽0,\\ g_{2}\left(X\right)=-x_{1}^{2}-x_{2}^{2}+2\cos135^{{}^{\circ}}x_{1}x_{2}-{\left(l_{4}+l_{1}\right)}^{2}⩽0. \end{array}\right. \end{array}$$

Using matlab to optimize the design, the results are as follows:

Relative length of connecting rod *l*_2_/*l*_1_ = 14.7497.

Relative length of rocker *l*_3_/*l*_1_ = 1.7039.

Combined with the overall size of the mechanism, take the length of the crank *l*_1_ = 8 and the length of the frame *l*_4_ = 120, and according to the matlab optimization design results, the connecting rod length and the rocker length can be obtained:

(27) $$\begin{array}{c} \left\{\begin{array}{c} l_{3}=14.7497\times 8\approx 118,\\ l_{4}=1.7039\times 8\approx 13.63. \end{array}\right. \end{array}$$

The kinematics simulation of the crank and rocker mechanism is performed, and the output angle function is shown in Figure 26.

Fitting result:

(28) $$\begin{array}{c} f\left(x\right)=35.65\sin\left(2\pi x-1.677\right)+102.9. \end{array}$$

It can be seen that the output angle function of the mechanism fits well with the objective function.

## 4. Conclusions

In this paper, a theoretical model of the interaction between the seahorse's dorsal fin and seawater is firstly carried out, and a fluid-structure coupling model suitable for this subject is derived, and then, a simulation model of the seahorse's dorsal fin and seawater is established based on the fluid-structure coupling theory and the physical properties of seawater. And refer to the Fluent database for parameter matching. Taking a certain working condition as an example, the interaction process between the seahorse's dorsal fin and the sea is analyzed, and the pressure distribution on the surface of the seahorse's dorsal fin and the flow field around it during the undulatory motion of the seahorse's dorsal fin is obtained through data postprocessing. Then, using the controlled variable method, keeping other variables the same, the influence of the swing frequency, wavelength, and amplitude of the seahorse's dorsal fin on the instantaneous force and average force in various directions of the seahorse's dorsal fin during the undulatory motion is studied, and the swing frequency, wavelength, and amplitude of the seahorse's dorsal fin are summarized. For the influence of the instantaneous force and the average force on the seahorse's dorsal fin in various directions during undulatory motion, finally, an optimal design method is used to design a seahorse-like dorsal fin undulatory motion mechanism, which has important guiding significance for the development of new underwater vehicle research and the miniaturization of the vehicle.

## Figures and Tables

**Figure 1:** Some types of seahorse's samples.

**Figure 2:** Coordinate system.

**Figure 3:** (a) Point cloud import to Solidworks. (b) Generated physical model of the dorsal fin.

**Figure 4:** Meshing diagram in ICEM.

**Figure 5:** Surface pressure distribution on the dorsal fin.

**Figure 6:** Section position.

**Figure 7:** Pressure distribution diagram of cross-sectional flow field.

**Figure 8:** Section position.

**Figure 9:** Cross-sectional flow field pressure distribution.

**Figure 10:** (a) *x*-direction force on the dorsal fin at different frequencies. (b) The relationship between amplitude of force and frequency. (c) The relationship between average value of force and frequency.

**Figure 11:** (a) *y*-direction force on the dorsal fin at different frequencies. (b) The relationship between amplitude of force and frequency. (c) The relationship between average value of force and frequency.

**Figure 12:** (a) *z*-direction force on the dorsal fin at different frequencies. (b) The relationship between amplitude of force and frequency. (c) The relationship between average value of force and frequency.

**Figure 13:** Frequency dependence of phase-averaged net thrust and power for (d). (a, b) Position of the leading edge *y*_LE_. (c, d) Net thrust (c) and power (d). Frequencies: ●: *f* = 0.5 Hz; ■: 1.4 Hz; ◊: 2.6 Hz; ×: 3.5 Hz.

**Figure 14:** *x*-direction force on the dorsal fin at different wavelengths.

**Figure 15:** *y*-direction force on the dorsal fin at different wavelengths.

**Figure 16:** *z*-direction force on the dorsal fin at different wavelengths.

**Figure 17:** *x*-direction force on the dorsal fin at different swing amplitudes.

**Figure 18:** *y*-direction force on the dorsal fin at different swing amplitudes.

**Figure 19:** *z*-direction force on the dorsal fin at different swing amplitude.

**Figure 20:** Mechanism assembly drawing.

**Figure 21:** Crankshaft components: (a) the left part; (b) the middle part; (c) the right part.

**Figure 22:** Right limit position of the joystick.

**Figure 23:** Different ranges of crank input angle correspond to rocker output angle.

**Figure 24:** Maximum and minimum transmission angle position of the mechanism.

**Figure 25:** Constraint planning area.

**Figure 26:** Crank-rocker output angle simulation.

**Table 1:** The number of fins and dorsal fin length of some types of seahorse.

Species	Amount of dorsal fins	Dorsal fin length				
		0~5	5~10	10~15	15~20	20~25
Big-belly seahorse	27–28					√
West African seahorse	17–18				√	
Narrow-bellied seahorse	17–19				√	
Barbour's seahorse	16–22				√	
Bargibanti's seahorse	13–15	√				
Réunion seahorse	16–18				√	
Short-snouted seahorse	20–21		√			
Giraffe seahorse	19–22			√		
Knysna seahorse	16–18				√	
Tiger tail seahorse	17–19			√		
Crowned seahorse	14		√			
Denise's pygmy seahorse	14	√				
Lined seahorse	18–19			√		
Fisher's seahorse	17–18		√			
Sea pony	14–17		√			

**Table 2:** Model boundary parameters.

Boundary name	Boundary type
Above surface	Wall
Below surface	Wall
Left surface	Wall
Right surface	Wall
Front surface	Wall
Behind surface	Wall
Inlet	Velocity-inlet
Outlet	Pressure-outlet

**Table 3:** Fluent simulation preset parameters.

Parameter	Prevalue
Solver	Pressure-based
Time	Transient
Turbulence model	SST
Pressure-velocity coupling	PISO
Transient formulation	First-order implicit
Other term spatial discretization	First-order upwind
Time step size	0.001 s/0.0001 s/0.00003 s
Number of time steps	4000

**Table 4:** *x*-direction force parameter values of the dorsal fin at different frequencies.

Parameter	*a*	*b*	*c*	*d*
Frequency				
1 Hz	-0.0274	1.02	-0.1266	-0.0016
10 Hz	-3.038	10.42	-0.2721	-0.1448
35 Hz	-36.51	36.16	-0.0187	-5.132
50 Hz	-84.58	51.59	-0.1224	-4.175
100 Hz	-283.7	104.9	-0.3844	-6.922

**Table 5:** *y*-direction force parameter values of the dorsal fin at different frequencies.

Parameter	*a*	*b*	*c*	*d*
Frequency				
1 Hz	-0.027	2.003	1.714	-0.2349
10 Hz	-2.769	20.13	1.600	-23.59
35 Hz	-33.06	73.5	1.919	-285.7
50 Hz	-70.69	100.5	1.667	-585
100 Hz	-276.1	201.3	1.612	-2346

**Table 6:** *z*-direction force parameter values of the dorsal fin at different frequencies.

Parameter	*a*	*b*	*c*	*d*
Frequency				
1 Hz	-0.0594	2.004	-0.0411	-0.4454
10 Hz	-5.995	19.99	0.1282	-46.41
35 Hz	-71.04	73.5	0.0686	-573.4
50 Hz	-146.7	100	0.1183	-1173
100 Hz	-583.2	200.4	0.0136	-4688

**Table 7:** *x*-direction force parameter values of the dorsal fin at different wavelengths.

Parameter	*a*	*b*	*c*	*d*
Wavelength				
133 mm	-3.637	10.05	0.3407	-0.0742
200 mm	-3.038	10.42	-0.2721	-0.1448
400 mm	-17.4	10.03	-2.1592	-0.7686

**Table 8:** *y*-direction force parameter values of the dorsal fin at different wavelengths.

Parameter	*a*	*b*	*c*	*d*
Wavelength				
133 mm	-1.556	20.12	1.5236	-13.85
200 mm	-2.77	20.13	1.5946	-23.59
400 mm	-2.636	19.97	2.336	-50.11

**Table 9:** *z*-direction force parameter values of the dorsal fin at different wavelengths.

Parameter	*a*	*b*	*c*	*d*
Wavelength				
133 mm	-4.735	20	0.07619	-27.15
200 mm	-5.995	19.99	0.1235	-46.41
400 mm	-4.671	19.93	-0.1782	-69.39

**Table 10:** *x*-direction force parameter values of the dorsal fin at different swing amplitudes.

Parameter	*a*	*b*	*c*	*d*
Amplitude				
*π*/12	-3.552	9.885	0.3358	-0.01746
*π*/6	-4.124	9.983	0.4201	-0.1871
*π*/6	-3.038	10.42	-0.2722	-0.1448

**Table 11:** *y*-direction force parameter values of the dorsal fin at different swing amplitude.

Parameter	*a*	*b*	*c*	*d*
Amplitude				
*π*/12	-0.5752	20.1	1.7978	-6.333
*π*/6	-2.142	20.04	1.9166	-20.42
*π*/5	-2.77	20.13	1.5946	-23.59

**Table 12:** *z*-direction force parameter values of the dorsal fin at different swing amplitudes.

Parameter	*a*	*b*	*c*	*d*
Amplitude				
*π*/12	-1.442	19.99	0.1344	-9.263
*π*/6	-4.833	19.99	0.1575	-33.73
*π*/6	-5.995	19.99	0.1235	-46.41

## Data Availability

The data used to support the findings of this study are included within the article.

## References

[1] Koldewey H. J., Martin-Smith K. M. (2010). A global review of seahorse aquaculture. *Aquaculture*.

[2] Job S. D., Do H. H., Meeuwig J. J., Hall H. J. (2002). Culturing the oceanic seahorse, _Hippocampus kuda_. *Aquaculture*.

[3] Olivotto I., Avella M. A., Sampaolesi G., Piccinetti C. C., Ruiz P. N., Carnevali O. (2008). Breeding and rearing the longsnout seahorse _Hippocampus reidi_ : rearing and feeding studies. *Aquaculture*.

[4] Woods C. M. (2002). Natural diet of the seahorseHippocampus abdominalis. *New Zealand Journal of Marine and Freshwater Research*.

[5] Lin Q., Fan S., Zhang Y. (2016). The seahorse genome and the evolution of its specialized morphology. *Nature*.

[6] Blake R. W. (1979). The swimming of the mandarin fishSynchropus picturatus(Callionyiidae: Teleostei). *Journal of the Marine Biological Association of the United Kingdom*.

[7] Blake R. W. (1976). On seahorse locomotion. *Journal of the Marine Biological Association of the United Kingdom*.

[8] Lighthill J., Blake R. (1990). Biofluiddynamics of balistiform and gymnotiform locomotion. Part 1. Biological background, and analysis by elongated-body theory. *Journal of Fluid Mechanics*.

[9] Consi T. R., Seifert P. A., Triantafyllou M. S., Edelman E. R. (2001). The dorsal fin engine of the seahorse (Hippocampus sp.). *Journal of Morphology*.

[10] Sfakiotakis M., Laue D. M., Davies B. C. An experimental undulating-fin device using the parallel bellows actuator.

[11] Breder C. M., Edgerton H. E. (1942). An analysis of the locomotion of the seahorse, Hippocampus, by means of high speed cinematography. *Annals of the New York Academy of Sciences*.

[12] Ashley-ross M. A. (2002). Mechanical properties of the dorsal fin muscle of seahorse (Hippocampus) and pipefish (Syngnathus). *Journal of Experimental Zoology*.

[13] Wei W., Quan X., Cao H. (2021). Research on the rapid closing jet mechanism of pistol shrimp’s claws based on fluid dynamic grid. *Mathematical Problems in Engineering*.

[14] Lourie S. A., Foster S. J., Cooper E. W., Vincent A. C. (2004). A guide to the identification of seahorses. *Project Seahorse and TRAFFIC North America*.

[15] Quinn D. B., Lauder G. V., Smits A. J. (2014). Scaling the propulsive performance of heaving flexible panels. *Journal of Fluid Mechanics*.

